# Dermokine mutations contribute to epithelial-mesenchymal transition and advanced melanoma through ERK/MAPK pathways

**DOI:** 10.1371/journal.pone.0285806

**Published:** 2023-07-11

**Authors:** Wenqiong Ma, Zexiu Wu, Mazaher Maghsoudloo, Iqra Ijaz, Marzieh Dehghan Shasaltaneh, Yuqin Zhang, Qiao Weng, Junjiang Fu, Saber Imani, Qing Lian Wen

**Affiliations:** 1 Department of Oncology, The Affiliated Hospital of Southwest Medical University, Luzhou, Sichuan, China; 2 Faculty of Advanced Science and Technology, Department of Genetics, Tehran Medical Sciences, Islamic Azad University, Tehran, Iran; 3 The Center of Research and Training for Occupational Technical Safety and Health, Tehran, Iran; 4 Sichuan Provincial Center for Gynecological and Breast Diseases, Southwest Medical University, Luzhou, Sichuan, China; 5 Faculty of Science, Department of Biology, University of Zanjan, Zanjan, Iran; 6 Department of Obstetrics & Gynecology, Nanjing Drum Tower Hospital, The Affiliated Hospital of Nanjing University Medical School, Nanjing, China; 7 Key Laboratory of Epigenetics and Oncology, The Research Center for Preclinical Medicine, Southwest Medical University, Luzhou, Sichuan, China; 8 Shulan International Medical College, Zhejiang Shuren University, Hangzhou, Zhejiang, China; University of Crete, GREECE

## Abstract

To discover vulnerabilities associated with dermokine (DMKN) as a new trigger of the epithelial-mesenchymal transition (EMT) -driven melanoma, we undertook a genome-wide genetic screening using transgenic. Here, we showed that DMKN expression could be constitutively increased in human malignant melanoma (MM) and that this correlates with poor overall survival in melanoma patients, especially in BRAF-mutated MM samples. Furthermore, *in vitro*, knockdown of DMKN inhibited the cell proliferation, migration, invasion, and apoptosis of MM cancer cells by the activation of ERK/MAPK signaling pathways and regulator of STAT3 in downstream molecular. By interrogating the in vitro melanoma dataset and characterization of advanced melanoma samples, we found that DMKN downregulated the EMT-like transcriptional program by disrupting EMT cortical actin, increasing the expression of epithelial markers, and decreasing the expression of mesenchymal markers. In addition, whole exome sequencing was presented with p.E69D and p.V91A DMKN mutations as a novel somatic loss of function mutations in those patients. Moreover, our purposeful proof-of-principle modeled the interaction of ERK with p.E69D and p.V91A DMKN mutations in the ERK-MAPK kinas signaling that may be naturally associated with triggering the EMT during melanomagenesis. Altogether, these findings provide preclinical evidence for the role of DMKN in shaping the EMT-like melanoma phenotype and introduced DMKN as a new exceptional responder for personalized MM therapy.

## Introduction

Malignant melanoma (MM) is a deadly invasive melanoma tumor with an increasing incidence worldwide, especially in light-skinned populations like China [1,2]. The MM is ranked as the highest tumor mutation burden cancer among solid tumors, with many new alterations in pathways controlling cell proliferation, differentiation, and survival [3,4]. Compared to other forms of melanoma cancer, MM is not fully curable even with early-stage diagnosis; so there is unmet biomedical research needed for the right undersetting of the mechanisms of tumors and the development of novel therapeutics [5]. From this view, the National Cancer Institute runs many exceptional responders pilot clinical trials to analyze different molecular subtypes of the MM tissue to determine whether certain molecular features can predict responses to molecular targeted and immunotherapy drugs [3,5].

It is now widely accepted that epithelial-mesenchymal-transition (EMT) is the main pathway during the switching of melanocytes between differentiated and invasive states, resulting in a high rate of metastasis and drug resistance [6]. Our pan-analyzing of melanoma samples by large-scale weighted gene co-expression network classified that during melanomagenesis, up-regulation of EMT- transcription factors contribute to vasculogenic mimicry (VM)-forming process, resulting in the resistance of anti-angiogenic and anti-vascular therapies for malignant tumor endothelial cells [7,8]. Therefore, transcriptome profiling of EMT/VM-mediated therapeutic resistance samples could be a valuable strategy for finding exceptional responders for the personalized melanoma therapy [9,10].

We recently boarded on a find for novel VM/EMT-targeted therapies genes that are differentially regulated during melanomagenesis. One such gene identified was determined to be identical to a recently reported skin-specific genes gene, phosphatidylserine-specific phospholipase A1-alpha and dermokine (DMKN) that contribute to melanomagenesis by triggering the EMT signaling pathway and VM formation [11,12]. These genes transcriptionally can be used as promising biomarkers for exceptional responders in the targeted melanoma therapy [12]. The DMKN is an unknown proinflammatory glycoprotein with different isoforms α, β, δ, and γ, acts as a soluble regulator of keratinocyte differentiation in inflammatory skin disorders [13,14]. Different isoforms of DMKN have different regulation patterns in the melanoma [13]. The DMKN-β is suggested to impair ERK’s phosphorylation in keratinocytes or early-stage skin tumor cells [15]. Recently has been reported that DMKN-β/γ, a dimmer isoform of DMKN by shared promoter expression patterns, is highly expressed in malignant tumors of pancreatic carcinoma and colorectal cancer [16,17]. The *in vivo* and *in vitro* finding indicated that DMKN contributes to cancer cell proliferation, migration, and invasion by triggering the EMT signaling pathway [18]. Despite numerous experimental studies, the prognostic values and downstream molecular function of the DMKN among EMT-driven melanoma remain unknown.

To understand vulnerabilities associated with DMKN that trigger the EMT signaling pathway and VM formation to promote melanomagenesis, we undertook a genome-wide genetic screening using transgenic. Here, we investigated the role of DMKN in advanced melanoma cells and showed that DMKN expression could be constitutively increased in advanced human melanomas and that this correlates with poor overall survival. By mimicking *in vitro* constitutive expression models, we report that DMKN contributes to melanoma cell growth, migration, and apoptosis. Furthermore, the knockdown of DMKN led to a significant decrease in many metastasized features and the formation of the VM, through ERK/MAPK pathways. These findings reveal an essential role for DMKN in melanomagenesis and highlight the role of DMKN as a new exceptional responder for personalized melanoma therapy.

## Materials and methods

### Ethics statement

This study was approved by the “Ethics Review Board” of the Affiliated Hospital of Southwest Medical University (No. KY2019041). Additionally, all clinical assessments were processed according to the local Ethics Committee guidelines of the Pathology and Surgery Department at the Affiliated Hospital of Southwest Medical University, Sichuan, China. Written informed consent that conformed to the tenets of the Declaration of Helsinki (1983 Revision) was obtained from all participants or their guardians for use of their clinical and pathology information, before the study. The authors had access to information that could identify individual participants during or after data collection.

### Cell lines and cell culture

Human advanced melanoma cell lines C8161, MUM-8B, SK-MEL-28, and A375, were purchased from American Type Culture Collection (ATCC, Manassas, VA, United States). All Cell lines were cultured in Dulbecco’s Modified Eagle’s medium (DMEM) supplemented with 10% fetal calf serum (Thermo Fisher Scientific, Waltham, MA, USA) and 1% penicillin-streptomycin (Sigma-Aldrich, St Louis, MO, USA) [19] in a humidified atmosphere of 5% CO_2_ at 37°C. The cell lines were regularly tested for mycoplasma contamination and confirmed mycoplasma negative before using in the study.

### Patients and clinical assessment

In total, 31 adult patients with advanced melanoma were enrolled, diagnosed, and treated in the Affiliated Hospital of Southwest Medical University, Luzhou, China, from September 2019 to September 2020. The pTNM Union for International Cancer Control (UICC) pathological staging criteria and World Health Organization (WHO) guidelines were used for diagnosis. The tissue specimens from the subjects with melanoma stage II-III in primary and III-IV were collected. Our database covers the histopathologic variables and the demographics of all the subjects included in the study. The fluorine-18-fluorodeoxyglucose positron emission tomography/computed tomography (^18^F-FDG PET/CT) imaging was utilized to assess and confirm the metastatic status; AJCC 8th edition was used for disease staging. All the included patients were clinically stable before inclusion in the study; cases with alongside comorbidities were excluded. Patients underwent standard treatments based on the practice of each treating physician. Table 1 shows the demographics and baseline clinical-philological characteristics of included subjects.

**Table 1:** Baseline clinic-pathological characteristics and dermokine (DMKN) expression in 31 MM cancer specimens.

Variable	No.	DMKN			
		mRNA level*	P-value	Protein level**	P-value
Gender					
Female	15	0.18 ± 0.05	0.731	33.35 ± 4.8	0.483
Male	16	0.16 ± 0.06		47.7 ± 5.7	
Age					
> = 60	19	0.22 ± 0.06	0.035	47.37 ± 5.08	0.042
< 60	12	0.09 ± 0.02		30.17 ± 4.82	
TNM stage					
II-III	12	0.07 ± 0.02	0.032	35.32 ± 3.92	0.041
IIIB-IV	19	0.22 ± 0.05		49.25 ± 6.22	
Anatomic location					
Face	3	0.15 ± 0.04	0.585	33.34 ± 9.91	0.323
Trunk and neck	2	0.09 ± 0.02		24.61 ± 2.51	
Upper limb and shoulder	2	0.08 ± 0.01		20.32 ± 6.01	
Lower limb and hip	19	0.15 ± 0.04		42.89 ± 5.02	
NA	5	0.30 ± 0.13		51.61 ± 9.67	
Pathology type					
Superficial spreading	16	0.19 ± 0.01	0.632	52.80 ± 11.54	0.117
Nodular	8	0.14 ± 0.02		50.03 ± 9.43	
Acral lentiginous	5	0.09 ± 0.06		38.70 ± 6.71	
Others	2	0.11 ± 0.01		38.44 ± 2.73	
Differentiation					
Poorly or none	9	0.08 ± 0.13	0.021	42.02 ± 8.05	0.032
Well or moderately	22	0.19 ± 0.21		60.12 ± 9.32	
Chemotherapy					
Yes	10	0.24 ± 0.08	0.816	33.75 ± 6.61	0.923
No	21	0.13 ± 0.04		44.05 ± 4.73	
Radiotherapy					
Yes	7	0.23 ± 0.11	0.398	39.58 ± 6.22	0.219
No	24	0.16 ± 0.04		41.05 ± 4.75	

Data are presented as mean ± SD for all others.

Patients were categorized according to the World Health Organization (WHO) guidelines and the pTNM Union for International Cancer Control (UICC) ‎pathological staging criteria.

Abbreviations: DMKN, dermokine; NA, Not applicable or not available; TNM, Tumor, node, metastasis (TNM) staging system.

* The expression of mRNA in advanced melanoma tissues was measured using real-time PCR analysis (qRT-PCR) and was normalized to that of the 18SRNA housekeeping gene using comparative Ct.

** The protein levels were quantified by immunobiological staining in tissue samples.

### RNA isolation and quantitative real-time PCR

Total RNA by Trizol reagent (Takara, Dalian, China) was isolated from frozen biopsies and melanoma cell lines following the manufacturer’s instructions. The qRT-PCR was carried out by the established techniques as previously described in [20]; to measure and evaluate the expression of the *dmkn* gene in all the samples. The *DMKN*, Foster City, CA), and using the comparative Ct method, the gene expression was obtained by normalizing to the GAPDH housekeeping gene [21,22]. S1 Table lists the primer sequences employed in this study.

### Immunohistochemistry staining

Immunohistochemistry was performed as described previously. Human melanoma tissue biopsies obtained at different stages were cut into sections and used for the immunohistochemical staining according to established protocols. DMKN was immunostained as previously described, using the streptavidin-biotin alkaline phosphatase complex technique by the Vectastain ABC-AP standard kit (Vector Laboratories; Burlingame, CA) [23–25]. Briefly, after dehydration, the antigenic epitopes were extracted from 5-μM sections using citrate buffer at pH 6.0 and microwaved for the 90s at high temperatures. Hydrogen peroxide (1%, 30 min at RT) plus methanol was used to quench endogenous peroxidase; and 2% normal mouse serum (Santa Cruz Biotechnology, Santa Cruz, CA) and levamisole (Vector Laboratories, Burlingame, CA) were used to inhibit unspecific antibody binding and quench the endogenous alkaline phosphatase for 30 min at RT, respectively. Samples were incubated with primary antibodies based on relevant concentrations according to the manufacturer’s guidelines (Vector Laboratories; Burlingame, CA) and subsequently incubated with biotinylated secondary antibodies after washing with phosphate-buffered saline (PBS) samples in a humid chamber for 10 minutes; primary and secondary antibodies are listed in S2 Table. Antibody staining was detected using the Vector Red alkaline phosphatase substrate kit (Vector Laboratories) and an avidin-biotin alkaline phosphatase complex (1:400 Promega, Madison, WI). Before being used for TMAs, all primary antibodies were titrated, and their specificity was tested using negative controls (Tris-buffered saline, normal preimmune rabbit IgG, and normal mouse IgG). Measurements and image acquisition were done in a blinded fashion using coded patient samples by (M.W. and M.Z.). Images for positive DMKN expression of samples were acquired on three different tumor stages at 50× and 100× magnification. The proportion of DMKN positive expression was calculated as the area of DMKN positive staining/the total area under a high magnification field of vision. DMKN immunostaining intensity was classified into negative-to-weak, moderate, and strong. All sections were seen using a Zeiss Axioplan 2 microscope, and photographs were taken on a Windows NT workstation and processed using Zeiss Axiovision software (Zeiss; New York, NY).

### Transduction with DMKN shRNA

All melanoma cell lines were transfected with NC or shDMKN (KD) plasmids purchased from GeneCopoeia Co. (GeneCopoeia Inc., MA, USA) as previously described by [26]. Twenty-four hours before transduction, the cell lines were plated with 1×10^5^ cells per well in 24-well plates containing 2ml medium (Qiagen, Hilden, Germany). Next, the medium was replaced with a 1ml shRNA lentivirus-containing medium in the presence of 8 μg/ml polybrene, according to manufactures instructions. After 12 hours of incubation, infected cells were chosen by adding 2 gml-1 Puromycin (Jena Bioscience, Jena, Germany) until no more live cells were present in a control plate that had not been transduced. The expanded single-cell clone transfection efficiency was confirmed with qRT-PCR and Western blot analyses.

### Transwell invasion assay

Corning Costar 24-well Transwell cell culture inserts with 6.5 mm diameter polycarbonate filters (8μM pore size, Corning, NY, USA) covered in 35 μL High Concentration Corning Matrigel Matrix (Becton, Dickinson, and Company, USA) was used to perform the invasion assay (Becton, Dickinson, and Company, USA) as described previously [25]. The inserts seeded with 5×10^4^ cells on the top of the chamber containing 1% FBS were allowed to invade for 24 h at 37°C. The PBS was used to wash chambers, and the fixed cells were treated with methanol for 20 min and then stained with Giemsa stain for 15 min. For examination, the invaded stained cells were manually counted in 5 randomly chosen fields, and representative photos were taken using an inverted microscope (Olympus Cor., Tokyo, Japan).

### Tumor metastasis assay *in vivo*

Melanoma C8161 and MUM-2B cell lines 5×10^4^ transfected NC or shDMKN were used for wound healing assay to check cell migration status as previously described by [27]. A sterile 200- μL pipette tip was used to generate scratches in the 90% confluent cell monolayer, after which the cells were rinsed with 3x PBS and grown at 37°C for 24 hours in a serum-free medium. At 0–24 h of induced injury, cell migration was assessed with a phase-contrast microscope (Olympus Cor., Tokyo, Japan), and the software ImageJ Wound Healing Tool plug-in was used to determine the migratory discrepancies.

### Western blot analysis

Inkblot analysis RIPA lysis buffer (Roche, Diagnostics, Mannheim, Germany) was used to correct the total cell lysate of advanced melanoma cell lines and biopsies of human melanoma tissues (Roche, Diagnostics, Mannheim, Germany). The polyacrylamide gel electrophoresis SDS/PAGE was used to resolve whole cell extracts, which were then moved to immobilon PVDF membrane and blocked with 5% bovine serum albumin for 30 min at RT. An improved chemiluminescence detection technique was used to identify the proteins of interest in immunoblots following incubation with primary antibodies. The antibodies utilized in western blotting are listed in S2 Table.

### Cell cycle analysis

The Cell cycle distribution between NC or shDMKN (KD) in C8161 and MUM-8B cells was performed as described earlier (49). The Cell Cycle Staining Kit, the PI/RNase staining buffer (BD Biosciences, CA, USA) was used in flow cytometry to determine the cell cycle, and ModFit LT2.0 software (Verity Software House, Topsham, ME, USA) was used for data analysis.

### Proliferation, cell migration, and invasion assays

Colony formation assays were implemented to examine the effect of DMKN on the proliferation of advanced melanoma cells. The cells were recovered in regular media for ten days, and colonies were counted. Real-time detection cell index of C8161 and MUM-8B with NC or shDMKN was analyzed as previously [20,28]. A real-time cell analyzer (xCELLigence RTCA DP, Roche, Germany) was used to analyze cell proliferation/growth index, migration, and invasion.

### Whole genome amplification (WGA) analysis

The MALBAC Single Cell Whole genome amplification Kit (cat. no. YK001A; Yikon Genomics, Inc.) was used for WGA of the advanced melanoma cell lines C8161, MUM-2B, and SK-MEL-28; carried out both before and after DMKN knockdown [29]. Advanced melanoma cell lines were subjected to the whole genome and targeted exome sequencing to check the knockdown expression of DMKN. WGS (30x) was performed to see the chromosomal breakpoint junctions and check the ratio of somatic point mutation variants, and the 10x WGS analyses were carried out between the shDMKN and NC control in the C8161 cells.

### Whole genome library preparation and sequencing

The Illumina paired-end libraries (Illumina, Inc.) techniques were used to detect and design the entire genome library and sequencing, as previously explained [30]. The amplified DNA (900 ng to 1 μg) from the advanced melanoma cell lines C8161, MUM-2B, and SK-MEL-28 was sheared into fragments of about 300 bp using a Covaris E220 system(Covaris Inc.). An aliquot of adaptor-ligated DNA was generated to use in the enrichment qPCR to establish the adaptor for Illumina PE sequencing. The pooled DNA (600 ng) from four barcoded libraries was utilized for hybridization and post-hybridization amplification according to the manufacturer’s instructions (SureSelectXT Target Enrichment System for Illumina Paired-End Sequencing Library; Illumina, Inc.). The results of the PCR amplification of cell lines were quality confirmed, and Illumina HiSeq 2000 (Illumina, Inc.) was used for WGS, with an average coverage depth of between 10x and 30x.

### *In silico* mutation analysis

The damaging effects of pathogenic mutations p.E69D and p.V91A in the DMKN protein functions were assessed *in silico* using online web servers Mutation Taster (http://www.mutationtaster.org/) [31], Polymorphism Phenotyping version 2 (PolyPhen-2, http://genetics.bwh.harvard.edu/pph2/) [31], SIFT (http://sift.jcvi.org/) [32], Have Your Protein Explained (HOPE) [33], and PANTHER (http://www.pantherdb.org/tools/csnpScoreForm.jsp) programs [34]. For SIFT, the functional impact of the mutation was described as "tolerated" or "damaging," whereas for Mutation Taster, it was labeled as "disease-causing" or "polymorphism." Following the classification system PolyPhen-2, the function of human proteins can be classified as "benign," "potentially detrimental," "probably damaging," or "unknown." I-Mutant3.0 was employed based on the stability predictors (DDG < 0: decrease stability, DDG > 0: increase stability) to forecast how stability would vary in response to mutations in the protein sequence or structure [35]. EBI/EMBL carried out paired alignment between the template and target. Additionally, by entering the data into the HomoloGene software of NCBI’s "Show Multiple Alignment" and Jalview software, the DMKN conservation in different organism genes was examined [36].

### Homological based modeling

The universal protein repository (http://www.uniprot.org) was used to download the sequence of the human p-ERK2 protein and the DMKN protein. The protein-protein interactions are known as the midpoint for all of the biochemical pathways involved in biological functions. The interactions were assessed in the high ambiguity driven protein-protein docking (HADDOCK) 2.2 program [37]. The protein structural calculations were guided by defining active residues based on the previous report [38], followed by selecting the structures with the least HADDOCK score and best binding site. Then, the program for automatically plotting protein-protein interactions (Ligplot-Dimplot, v 2.2.5) was applied to determine intermolecular contacts such as hydrogen bonds and non-bonded ones, and VMD was employed to visualize the model [39,40]. Our molecular simulations’ for DMKN were based on the template protein’s crystal structure (PDB Entry: S700672). Using Pymol software, a mutation of the nsSNPs E69D and V91A was produced *in silico* from the WT crystal structure [41]. The final modeled protein structure’s overall stereochemical quality was assessed using PROCHECK [42], ProSA-web (protein structure Analysis) [43], and QMEAN analysis [44].

### Genomic CNVs and gene set enrichment analysis

We used the standard probe to identify genomic copy number variations (CNVs) in the advanced melanoma cell lines C8161, MUM-2B, and SK-MEL-28 as developed by Zong et al. [45]. Using the publicly accessible online University of Santa Cruz (UCSC) database and Burrows-Wheeler Aligner v0.6.1 [46], the paired-end sequencing reads of each cell line were aligned with the Human Genome version 19 (hg19). The input and output files, as well as the submission of analyses for execution, were managed by the Firehose pipeline (level 4) [47]. ControlFreeC was used to detect single-nucleotide and CNVs across the genome of a single human cell [48]. In hidden Markov model-based calling algorithms (HMMs), the result is a binary array that indicates whether a single cancer cell has better coverage than normal leukocytes [49,50]. The hg19 serves as the reference genome; the copy number analysis was carried out using information from the Ginkgo dataset (http://qb.cshl.edu/ginkgo) and two R tools (HMM copy and DNA copy). Functional enrichment analysis was performed with an integrative method that discovers significantly enriched pathways, across multiple datasets such as BioCyc [51], KEGG [52], Reactome [53], GenMAPP [54], MSigDBBioCarta [55], PantherDB [56]. Enrichment tests were carried out at the arm level to determine whether chromosome arms had significantly gained or lost. The GSEA was additionally employed for a functional evaluation of the established disease pathways among cell lines that shared CNVs [57]. In light of this, we used R software (v3.3.1) pathway analyses to discover probable biological functional evaluation of shared CNVs [58].

### Statistics

The SPSS software version 21.0 (Chicago, Illinois, USA) was employed for statistical analysis. The software GraphPad Prism 5.0 was used to create each graph (GraphPad Software Inc., La Jolla, CA, USA). For *in vitro* quantitative data, the biological experiments were performed thrice. A Linear logistic regression analysis was conducted between DMKN and common diagnostic biomarkers of malignant melanoma, Ki67, p53, Melanin A, and S-100 in stage II-IV melanoma. Spearman’s rank correlation coefficient test was employed to determine the association between two variables. Variations were displayed as mean and SEM for each group. The Kaplan-Meier method uses the log-rank test to determine the possible relationship between DMKN expression and disease-free survival (DFS) of MM patients. Fisher’s exact test was used to assess the level of enrichment of mutations/aberrations that alter the pathway in the shDMKN (KD) group compared to the NC. P values < 0.05 were regarded as significant; individual P values and details of statistical analysis are also included in the figure captions.

## Results

### DMKN is overexpressed in advanced melanoma cell lines and correlated with the tumor grade and diagnostic biomarkers in MM specimens

The results of the previous studies represented that DMKN could be utilized as a reliable and distinctive biomarker among nevi- and primary-metastatic melanoma patients. In the present study, the function of DMKN, as well as its relationship with malignancy in melanoma cancer was examined by analyzing the mRNA and protein expression of DMKN-α, DMKN-β, and DMKN-β/γ in the aggressive amelanotic human melanoma cell line (C8161), uveal melanoma cell line (MUM-2B), and two other advanced melanoma cell lines (SK-MEL-28 and A375) (Fig 1A and 1B). The expression of DMKN significantly increased in all advanced melanoma cell lines, while no significant difference was observed in the A375 cell line. Additionally, DMKN-β/γ was highly expressed in advanced metastatic melanoma, similar to DMKN-β. The qRT-PCR and IHC methods were respectively applied to assess DMKN levels during melanogenesis in 31 MM samples. Given the simultaneous consideration of both gene and protein, DMKN levels were associated with tumor invasion (p = 0.034) and significantly elevated in the advected melanoma stage (Table 1). In terms of the frequency of DMKN, a significant rise was detected in distant metastatic tumors (50.44 ± 9.36) compared to the M0 distant metastatic ones (31.40 ± 13.13; p = 0.018) (Fig 1C). However, DMKN expression was not correlated to sex, age, and tumor differentiation (Table 1). The expression level of the different isoforms of DMKN is challengeable in a wide range of MM samples with various morphologies (Fig 1D). To verify the association between DMKN with a type of MM diagnostic biomarkers, a linear logistic regression analysis was employed to predict the accuracy of the DMKN expression detection between the different stages of MM samples (Fig 1E). The simultaneous consideration of the expression levels of both gene and protein suggested a positive correlation between relative DMKN levels with the routine diagnostic biomarkers of MM such as Melan-A (r = 0.054; p = 0.011), Ki67 (r = 0.08, p = 0.034), and BRAF (r = 0.012; p = 0.044). However, the relative DMKN levels were inversely correlated to P53 (r = -0.014; p = 0.021). Further, a significant correlation was observed between DMKN expression with the clinicopathological features of subjects with MM (Table 2). The higher DMKN levels were correlated with disease severity and metastatic lesions among the individuals with MM.

**Fig 1:** The cancerous role of DMKN in advanced melanoma. (A) Relative levels of DMKN-α, DMKN-β, and DMKN-β/γ mRNA expression in advanced melanoma cell lines. (B) DMKN protein level in advanced melanoma cell lines. (C-D) Quantification and representative immunobiological staining imaging of DMKN expression in tissue samples from different stages. (E) Linear logistic regression analysis between DMKN and routine diagnostic biomarkers (Ki67, p53, Melanin A, and S-100) in stage II/III melanoma (blue cycle) and stage III/IV melanoma (red cycle). (F) Disease-free survival (DFS) rate based on DMKN expression in 15 patients with low DMKN and 16 patients with high DMKN. (G) DMKN expression in advanced melanoma with different mutation stages (BRAF, NRAS) and EMT features. (H) Receiver operating characteristic curve for DMKN mRNA and protein expression in EMT+ MM group (blue line), NRAS mutant MM group (green line), and BRAF mutation group (red line). The diagnostic values were calculated based on DMKN mRNA expression and protein levels. Patients were categorized as low-DMKN when FC < 0.18 for DMKN mRNA expression and < 42.78 for protein DMKN levels. The grouping of western blot gel images was cropped from different parts of the same gel. The full-length gels are included in S1 Raw images. High DMKN is defined as FC ≥ 0.18 for DMKN mRNA expression and ≥ 42.78 for protein DMKN levels.

**Table 2:** The common oncogenic variables in the study of patients.

Oncogenic variable^#^	Melanoma patients	
	Primary^#^ (n = 12)	Metastasis (n = 19)
*DMKN*	35.32 ± 3.92	49.25 ± 6.22
*p53*	23.25 ± 3.35	58.32 ± 2.43 *
*Ki67*	40.12 ± 5.41	69.32 ± 10.11 *
*Melan-A*	41.12 ± 7.76	25.74 ± 12.8 *
*S-100*	32.04 ± 2.63	59.43 ± 1.06 *
*HMB-45*	28.75 ± 2.81	25.12 ± 2.81
*CK-8*	27.19 ± 8.33	30.14 ± 4.40
*SAM*	19.84 ± 0.65	24.24 ± 1.96

**Abbreviations:** DMKN, dermokine; p53, TP53 or tumor protein; melan-A, Melanoma Antigen Recognized by T cells; S-100, S100 calcium-binding protein B; HMB-45, human melanoma black 45; CK-8, cytokeratin-8; SAM, S-adenosylmethionine.

Data are presented as mean ± SD for all others.

* P < 0.05 and ** P < 0.001 vs metastasis group.

^#^The protein levels of the oncogenic genes were quantified by immunobiological staining in tissue samples.

^##^ Primary groups are stage II/III melanoma patients and metastasis is covered in stage III-IV melanoma patients.

### DMKN expression stratifies survival in human melanoma cancer

Finding an effective diagnostic strategy to detect MM can allow the development of a subsequent targeted therapy that can improve the prognostic outcomes and therapeutic approaches among advanced MM patients. In this regard, the subjects (n = 31) were categorized according to their DMKN levels (lower than, equal to, or higher than the mean expression of DMKN) to determine any possible relationship between DMKN expression with the DFS of the individuals with MM through using the Kaplan–Meier method and log-rank test (Fig 1F). Based on the immunobiological staining index, FC: 0.18 and 42.28 were considered for DMKN mRNA expression and protein DMKN levels, respectively. Given both DMKN mRNA and protein levels, patients were classified as either low-DMKN or high-DMKN. Low-DMKN patients had an FC value less than 0.18 for DMKN mRNA expression and a serum DMKN level greater than 42.78 μg/L, while high-DMKN patients had an FC value less than or equal to 0.18 for DMKN mRNA expression and a serum DMKN level equal to or greater than 42.78 μg/L. As expected, the subjects with melanoma with high-DMKN tumors had a significantly shorter DFS than those with low-DMKN tumors (three-year DFS rate: 66.2% vs 75.4%, *p  =* 0.03). This result indicated a worse prognosis among patients with high-DMKN tumors than those with low-DMKN tumors (*p  <* 0.05). Further, a depletion in DMKN in the epithelial cells led to an EMT and tumor progression. A question was raised can DMKN expression be used to differentiate a comma mutation type of MM-like BRAF/NRAS MM tumors from the EMT+ and epithelial subgroups of MM tumors (Fig 1G). Fig 1G demonstrates the Area Under the Curve (AUC) related to the Receiver Operating Characteristic (ROC) analysis of protein and mRNA levels in the various types of mutations. Correspondingly, a significant rise was found in DMKN expression in the MM with an EMT signature and BRAF/NRAS MM tumors (Fig 1H; *p  <* 0.05). Indeed, DMKN expression differentiated between the BRAF/NRAS MM tumor with the EMT+ subgroups of MM tumors. Furthermore, high DMKN expression was correlated with better therapy response and overall patient survival. Considering both DMKN mRNA and protein levels, the results of ANOVA among BRAF/NRAS mutated samples revealed the greater accuracy of DMKN for BRAF-MUT samples than the NRAS-MUT ones. Similarly, the high expression of DMKN was correlated with the EMT signature in the MM. The pooled sensitivity and specificity were more in the EMT+ subgroups of MM samples compared to the EMT- subgroups. The results represented a significant correlation between low DMKN expression and poor survival in these MM. The DMKN had the highest sensitivity, specificity, and AUC in EMT+ advanced melanoma, suggesting its usability as a marker to effectively predict and diagnose advanced BRAF-mutant and EMT+ melanoma cancer. In general, the high expression levels of DMKN were correlated with MM EMT signatures and poor survival among these cancer patients.

### DMKN knockdown slightly decelerates MM cell phenotype *in vitro*

The DMKN protein expression was analyzed in untransformed MM cells and various MM cell lines to investigate the role of DMKN in melanomagenesis. Due to the lack of common sequence regions in the DMKN-α, DMKN-β, and DMKN-β/γ, different short-hairpin RNA (shRNA)-gene silencing constructs were designed for all three isoforms (Table 3). Then, the most effective shRNA-DMKN was transduced to various MM cells, and the gene and protein expressions of DMKN were determined by using the qRT-PCR and Western blotting methods, respectively (S1 Fig). Regarding the C8161 and MUM-2B cell lines, the expression of DMKN-β/γ genes was almost completely lost in the DMKN-shRNA-transduced cells (shDMKN) compared to the lentivirus-scrambled control (NC) (Fig 2A and 2B). Accordingly, these cell lines were selected for future *in vivo* analysis. Upon transduction of the most effective shRNA-DMKN, we found that the expression of DMKN-β genes was almost completely lost in the C8161 and MUM-2B cell lines. These results indicate that DMKN-β is the main expressed isoform of DMKN in metastatic melanoma and therefore were selected for future in vivo analysis. Thus, in the rest of our paper, we refer to DMKN as the DMKN-β isoforms since these were the main isoforms expressed in metastatic melanoma cells and the focus of our study. We hope that this clarification will help readers to better understand the scope of our investigation and the significance of the DMKN-β isoforms in melanoma progression. The results of the initial invasive screening exhibited the effect of DMKN knockdown on the proliferation/viability of the C8161 cell line compared to the MUM-2B malignant one (Fig 2C and 2D). The results of time-course cell proliferation/viability measurement represented an effective reduction in the amount of DMKN (> 80%) at three and four days post-transfection with shDMKN in the C8161 and MUM-2B cells, respectively. Furthermore, the DMKN knockdown significantly suppressed the invasion of C8161 and MUM-2B cells compared to the LV-shNC-infected C8161 and MUM-2B cells (Fig 2E), as well as that of MM cells compared to the LV-shNC-infected MM ones.

**Fig 2:** DMKN knockdown inhibits proliferation and invasion in advanced melanoma cell lines. The *dmkn* gene (A) and protein (B) levels in DMKN-shRNA-transduced cells (shDMKN) compare to that in lentivirus-scrambled control (NC). Analysis of cell invasion by using a modified Boyden Chamber assay. in lentivirus control and DMKN-shRNA-transfected in the C8161 and MUM-2B cell lines. Microscopic picture of invaded cells (C) represents Bar graph (D) and the number of cells invaded the matrigel. (E) Relative cell viability of shDMKN (red line) or NC (black line) cells. Cell proliferation values are presented as the mean SEM of three independent tests. Values are as mean ± SEM, n = 3, **p < 0.001 for NC. The grouping of western blot gel cropped from different parts of the same gel. During the invasion assay, the leftover supernatants on the upper chamber of the transwell insert were collected from all the treatments of both cells.

**Table 3:** Sequences of shRNA vectors were prepared for this study.

Target gene	No.*	Start position**	Intrinsic Score^#^	5’ Seq.	Loop Seq.	3’- Seq.	Target Seq.	Reverse seq.	Full seq.
**DMKN-α**	NM_001352330.2	884	15.10	CCGG	CTCGAG	TTTTTG	GAGTTTCTCTGTGGAAATAAA	TTTATTTCCACAGAGAAACTC	5’-CCGGGAGTTTCTCTGTGGAAATAAACTCGAGTTTATTTCCACAGAGAAACTCTTTTTG-3’
**DMKN-β**	NM_001126056	258	14.20	UUGG	AUUUA	TTTTTG	GGAAAGCACTGGGACAAATAT	ATATTTGTCCCAGTGCTTTCC	5’-UUGGGGAAAGCACTGGGACAAATATAUUUAATATTTGTCCCAGTGCTTTCCTTTTTG-3’
**DMKN-β/γ**	NM_001035516.4	131	14.70	AAAA	GCAGAG	TTTTTG	CGATCAGAACTACAATTACAA	TTGTAATTGTAGTTCTGATCG	5’-AAAACGATCAGAACTACAATTACAAGCAGAGTTGTAATTGTAGTTCTGATCGTTTTTG-3’

Abbreviations: DMKN, dermokine; 5’ Seq., Sequence of the 5’ arm of the hairpin; Loop Seq., The sequence of the loop connecting the two arms of the hairpin; 3’- Seq., Sequence of the 3’ arm of the hairpin; Target Seq., Sequence of the target gene that the hairpin is designed to bind to reverse sequence; Reverse seq., Reverse complement sequence of the hairpin; Full seq., Complete sequence of the hairpin including both arms and the loop.

* Genbank accession number of cDNA and corresponding gene, available at http://www.ncbi.nlm.nih.gov/‎.

** Start position of hairpin’s match to the targetted transcript sequence (1-based).

^#^ Also called "original score", this assesses the target sequence for predicted clone ability and knockdown performance.

### Reduced DMKN expression inhibited invasion and migration in MM cells and induced cell cycle arrest

The effect of DMKN on MM migration and invasion was assessed through the transient transfection of shDMKN into the C8161 and MUM-2B cell lines, respectively (Fig 3). The results revealed that shDMKN failed to significantly inhibit cell proliferation in MM cells. Based on the *in vitro* wound-healing assay results, significantly less migration was detected in both C8161 and MUM-2B cells (Fig 3A). In the C8161 cells, the shDMKN exhibited the highest reduction in migration after 24 hr of cell culture (Fig 3B). In addition, the results of the migration assay in Boyden Chambers demonstrated that shDMKN decreased the migration of C8161 and MUM-2B cells (Fig 3C). After five days of culture, the DMKN knockdown diminished cell migration in the advanced melanoma cell lines. The mean fluorescence related to cell migration was 89.20 ± 32.24 in the C8161 cell line (control: 120.00 ± 45.21) and 117.20 ± 9.43 in the MUM-2B one (control: 124.05 ± 11.81), respectively (Fig 3D). Further, the real-time cell analyzer results indicated that shDMKN dependently inhibited the migration and invasive characteristics of C8161 cells (Fig 3E). The results related to the effect of DMKN on inhibiting the clonogenicity of C8161 and MUM-2B cells suggested a significant reduction in colony formation following the transient transfection of shDMKN into the cell lines, respectively (Fig 3F and 3G). Based on the results of cell cycle progression analysis in Fig 3H, shDMKN cells were arrested at the G0-G1 phase three days after DMKN transfection. Concurrently, the increased G0-G1 arrest and decreased G1-M phase were found in LV-shDMKN-infected C8161 cells with the G0-G1 ratio of 9.5 compared to the 0.45-fold for the NC controls (Fig 3I). Therefore, the mitotic arrest of tumor cells can be addressed as another potential mechanism by which DMKN may induce tumor growth. In general, the results represented that the expression of DMKN triggered cell invasion, migration, and clonogenicity in advanced melanoma.

**Fig 3:** DMKN knockdown reduced cell migration in advanced melanoma cell lines. (A) Scratch wound-healing assay of C8161 and MUM-8B cells transfected with GFP lentivirus (NC) or DMKN-shRNA (shDMKN). The movement of cells into the wounds was shown at 0 and 24 hrs after scratching (magnification: 10x). (B) The bar graph represents the number of cells that migrated into the scratched area. (C) Representative fluorescence microscopy photos in C8161 and MUM-8B cells transfected with NC or shDMKN within 5 days of treatment. (D) Bar graphs showing means fluorescence of migrating in C8161 and MUM-8B cells transfected with NC or shDMKN within 5 days of treatment. (E) Real-time detection cell index of C8161 and MUM-8B with NC or shDMKN in the xCELLigence real-time cell analysis. (F) Representative microscopic photos of the colony formation assays to examine the effect of DMKN on the proliferation of advanced melanoma cells. (G) The bar graph represents the number of cells that migrated into the scratched area. The cells were recovered in regular media for 10 days and colonies were counted. (H) Bar graphs showed the percentage of each cell cycle phase in C8161 and MUM-8B cells transfected with shDMKN or NT siRNAs for 3 days. (I) Representative percentage of each cell cycle phase in C8161 and MUM-8B cells transfected with shDMKN or NT siRNAs for 3 days. Expression of DMKN triggers cell cycle arrest and inhibits cell invasion in advanced melanoma cell lines. Values are as mean ± SEM, n = 3, **p < 0.001, ***p < 0.0001 for NC.

### Whole exome sequencing identifies somatic loss of function mutations in shDMKN-infected MM

The comparable WES was performed in the advanced melanoma cell lines (C8161, MUM-2B, and SK-MEL-28) before and after DMKN knockdown to determine the mutational landscape of DMKN during melanogenesis. These cell lines covered all of the known genetic subtypes of MM. Thus, an unbiased and integrated comprehensive genetic analysis, as well as *in vitro* functional analyses were conducted to validate the association pathways between the ShDMKN and NC (Figs 4A and S2). Extensive filtering and optimal-quality parameter thresholds for WGS analysis were robustly used to call high-confidence and Loss of Function (LoF) mutations between shDMKN and NC, respectively. Following the confirmation of targeted exome sequencing, 208 new LoF mutations between all three MM cell lines, 221 ones in shDMKN-C8161, 144 ones in shDMKN-MUM-2B, and 46 ones in shDMKN-SK-MEL-28 were recognized after comparing with the NC (Fig 4B and S3 Table). These genes included 286 (71%) genes with 252 high-confidence mutations (113 single-nucleotide variants (SNVs) and 139 INDELs) and 122 ones (29.9%) with 317 predicted low-confidence mutations (112 SNVs and 205 INDELs) (Fig 4C and 4D). After somatic mutation filtration, 120268 variants were set for further processing with maftools. A total of 95897 variants (601 unknown and 95296 silent) were removed during processing, and only 24371 somatic variants were considered by maftools for further analysis and reporting. As expected, SNV-polymorphism was the most abundant type (96.06%), among which SNP is more abundant than the transversions (Figs 4E and S3). As shown in Fig 4F, the mean number of variants per sample is ~7/2, and C > T (42%) and T > C (38%) are the most common classes of SNVs in the SNV transition. Furthermore, the results indicated a high mutation load of shDMKN-C8161 samples. The bottom right panel in Figs 4G and S4 reflects the barplot of the top 20 and 50 cancer-driver genes in the samples with a high number of mutations. The GSEA was employed for the functional assessment of the genes involved in melanomagenesis and cancer-driver genes. Table 4 compares the results of analyzing the most significantly enriched pathways of cancer-driver genes in the shDMKN-C8161 and GFP lentivirus (NC) control across multiple datasets such as BioCyc [51], KEGG [52], Reactome [53], GenMAPP [54], MSigDBBioCarta [55], PantherDB [56].

**Fig 4:** The whole genome and targeted exome sequencing results after the knockdown of DMKN in advanced melanoma cell lines. (A) Visualization of chromosomal breakpoint junctions between the shDMKN- C8161 and GFP lentivirus (NC) control. (B) The differentially expressed pathogenic genes with the largest fold changes between shDMKN-KD and NC in the different melanoma cell lines. (C) The ratio of somatically point mutation variants between shDMKN-KD and GFP lentivirus (NC) control in C8161 cells. The down panels above describe the variant classification (D), variant type (E), SNV class (F), and variant per sample in all shDMKN cell lines. (G) Top 20 frequently implicated genes out of the 221 genes mutated in the shDMKN-C8161 melanoma cell lines genome.

**Table 4:** Most significantly enriched pathways analysis of cancer driver genes in shDMKN lentivirus (KD) and GFP lentivirus (NC) control in C8161 cell.

	Pathway	Source*	p-value	Hit Count in Genome	Hit in Query List
**GFP lentivirus (NC) control**	HIV-I Nef: negative effector of Fas and TNF	MSigDB	0.0009	56	RB1,PRKCD,CDK11B
	Neurotrophin signaling pathway	MSigDB	0.0098	126	CAMK2G,PRKCD,TP53
	Cell cycle	MSigDB	0.0097	125	RB1,TP53,CDK7
	LKB1 signaling events	Reactome	0.0095	42	BRSK1,TP53
	Histamine H1 receptor mediated signaling pathway	PantherDB	0.0095	42	PRKCD,GNA11
	ATF-2 transcription factor network	Reactome	0.0093	55	NF1,PDGFRA,MMP2
	Cell cycle	GenMAPP, KEGG	0.0093	124	RB1,TP53,CDK7
	Melanoma	MSigDB	0.0093	68	NF1,RB1,PREX2,TP53
	Checkpoint Signaling in response to DNA damage	MSigDB	0.0092	13	RB1,TP53
	Neural Crest Cell Migration during Development	MSigDB	0.001	41	MMP2,MMP8
**DMKN-shRNA lentivirus (KD)**	Thromboxane A2 receptor signaling	MSigDB	0.00099	56	PRKCD,GNA11,RAC1
	HIV-I Nef: negative effector of Fas and TNF	MSigDB	0.00099	56	RB1,PRKCD,CDK11B
	RAC1/PAK1/p38/MMP2 Pathway	MSigDB	0.00099	69	TIE1,MMP2,TP53,RAC1
	Neurotrophin signaling pathway	MSigDB	0.00098	126	CAMK2G,PRKCD,TP53,RAC1
	Cell cycle	MSigDB	0.00096	125	RB1,TP53,CDK7
	LKB1 signaling events	Reactome	0.00095	42	BRSK1,TP53
	Histamine H1 receptor mediated signaling pathway	GenMAPP, PantherDB	0.00095	42	PRKCD,GNA11
	ATF-2 transcription factor network	Reactome	0.00094	55	NF1,PDGFRA,MMP2
	Cell cycle	GenMAPP, KEGG	0.00094	124	RB1,TP53,CDK7
	Pathways in cancer	MSigDB	0.00092	325	PDGFRA,RB1,MMP2,TP53,RAC1,RAC2

Abbreviations: GFP, Green Fluorescent Protein; NC, Negative Control; HIV-I, Human Immunodeficiency Virus type 1; Nef, Negative effector of Fas and TNF; RB1, Retinoblastoma 1; PRKCD, Protein kinase C delta; CDK11B, Cyclin-dependent kinase 11B; CAMK2G, Calcium/calmodulin-dependent protein kinase type II subunit gamma; TP53, Tumor protein p53; BRSK1, BR serine/threonine kinase 1; NF1, Neurofibromin 1; PDGFRA, Platelet-derived growth factor receptor alpha; MMP2, Matrix metalloproteinase-2; PREX2, Phosphatidylinositol-3,4,5-trisphosphate-dependent Rac exchange factor 2; MMP8, Matrix metalloproteinase-8; RAC1, Ras-related C3 botulinum toxin substrate 1; TIE1, Tyrosine kinase with immunoglobulin-like and EGF-like domains 1; RAC2, Ras-related C3 botulinum toxin substrate 2. The sources for functional enrichment analysis are MSigDB, Molecular Signatures Database; Reactome, a freely available, peer-reviewed pathway database; GenMAPP, Gene Map Annotator and Pathway Profiler; KEGG, Kyoto Encyclopedia of Genes and Genomes; PantherDB, Protein ANalysis THrough Evolutionary Relationships; BioCyc, a collection of Pathway/Genome Databases; MSigDBBioCarta, a subset of MSigDB containing pathway definitions from the BioCarta online resource.

* Functional enrichment analysis was performed with an integrative method that discovers significantly enriched pathways, across multiple datasets such as BioCyc [19], KEGG [20], Reactome [21], GenMAPP [22], MSigDBBioCarta [23], PantherDB [24].

The Copilot in Fig 5 illustrates the results of GSEA on the top 20 mutated genes in all three LV-shDMKN-infected MM cell lines. An oncoplot is a combination of gene- and sample-level summary, and patient clinical information, providing substrates for selecting potential oncogenes in the cancer cohort. In the present study, 86% of the top 100 frequently-mutated genes in this analysis were known cancer genes (Fig 5A and S4 Table). The most significant biological pathways related to melanomagenesis are sorted in Fig 5B. As displayed, the four common target pathways involve cell-cell communication, tight junction, collagen degradation, and melanoma. The p53 signaling, VEGF signaling, and G1-to-cell cycle control pathways with their response genes are higher in the LV-shDMKN-infected MM cell lines compared to the NC. This result may be partly attributed to the function of the DMKN in melanomagenesis. After the DMKN knockdown, the NF-1, BRAF, and TP53 oncogenes harbored mutations across the most enriched pathways (24%), reflecting their importance in melanomagenesis by triggering with the DMKND (Fig 5B). The most enriched functional cluster included three disease-associated oncogenes (NF-1, BRAF, and TP53) and three others acting in chromosome segregation, which is developmentally manifested as the intellectual growth of monocytes.

**Fig 5:** DMKN interactome is reprogrammed in MM cells. (A) The gene set enrichment heatmap indicates the mutation patterns of the top 20 most frequently implicated cancer driver genes with a high number of mutations in the shDMKN-C8161 melanoma cell lines genome. Each column represents an affected individual, and each row represents a gene. (B) Gene set enrichment analysis of most deregulated cellular processes among 984 genes carrying mutations/aberrations in the shDMKN (KD) group. The genes are halighlited in red color involved in melnomagesis. The p-value for each process represents the significance level for the enrichment of mutations/aberrations that affect this pathway in the DMKN-shRNA lentivirus (KD) group compared to the GFP lentivirus (NC) control and was calculated by two-sided Fisher’s exact test.

### DMKN induces EMT via the ERK/MAPK signaling pathway

The differential effects of various DMKNs on EMT and growth in the MM were further examined by retrovirally repressing the DMKN in the inherently epithelial-looking C8161 and MUM-2B cells, and evaluating the putative changes in cell morphology and other phenotypes (Fig 6). In the advanced MM, the characteristics of DMKN-repressed EMT were associated with the disruption of MET/EMT cortical actin, greater expression of epithelial markers (E-cadherin and ZO-1), and lower expression of mesenchymal markers (N-cadherin, vimentin, and Snail) (Fig 6A). These features were partially reverted following the DMKN knockdown in ShDMKN-C8161 compared to the NC control (Fig 6B), as well as the increased expression of epithelial (E-cadherin) and decreased expression of mesenchymal markers (Snail). However, vimentin and N-cadherin remained unchanged. Regarding both C8161 and MUM-2B cells, the DMKN significantly affected other EMT markers like Snail in knockdown (Fig 6B). Additionally, the effect of transfection with DMKN-shRNA lentivirus on the main oncogenic signaling pathways in the MM cells was studied to better understand the DMKN regulation of EMT.

**Fig 6:** Analysis of the oncogenic pathways regulated by DMKN. (A-B) the DMK disruption of MET/EMT cortical actin, increased expression of epithelial markers (E-cadherin), and decreased expression of mesenchymal markers (N-cadherin, Vimentin, and Snail). Expression of EMT-associated and oncogenic pathway proteins in DMKN-shRNA (KD), and GFP lentivirus (NC) were assayed in both gene (A) and protein levels (B). (C-D) ERK/MAPK signaling pathway was active with shDMKN downregulation as compared to NC in C8161 and MUM-2B MM cell lines. Expression of ERK/MAPK oncogenic pathway proteins in advanced melanoma cells transfected with either DMKN-shRNA (KD) or GFP lentivirus (NC) were assayed in both gene (C) and protein levels (D). The grouping of western blot gel is cropped from different parts of the gel. Whole-cell lysates (50–70 μg) were subjected to Western blotting analysis. GAPDH as loading control is shown with a representative blot. Values are as mean ± SEM, n = 3, **p < 0.001, ***p < 0.0001 for NC.

Despite a decline in the levels of the EMT and cell cycle-associated proteins identified previously, and reported MAPK/ERK1/2 downstream, the same signaling proteins were more phosphorylated in the KD than in the NC group (Fig 6C and 6D). The down-expression of DMKN resulted in reducing the activity of MMP2, MMP9, and VEGF, as well as enhancing that of the ERK1/2 and p-ERK1/2. Phospho-ERK1/2 was triggered via the STAT3 and AKT signaling as the main above-mentioned oncogenic pathways. Thus, more evaluations are needed to test whether DMKN serves as a regulator of STAT3 and downstream molecules. The results of further investigation suggested that the higher DMKN expression promoted cell growth, migration, and invasion of MM.

### Pathogenic mutations of the dmkn gene associated to melanomagenesis

To date, no disease-causing hotspot *DMKN* gene mutations have been reported in the available genotype-phenotype databases including the Human Gene Mutation Database (HGMD) [59] and Online Mendelian Inheritance in Man (OMIM) [60], as well as a database of Genotype and Phenotype (dbGAP) [61]. The present study characterized all disease-causing SNP mutation spectra in DMKN in the advanced melanoma cell lines (i.e., C8161, MUM-2B, and SK-MEL-28) (S5 Table). As shown, the nonsynonymous mutations of G > A are more widely observed and change highly conserved amino acids in DMKN. Following the *in silico* prediction pipeline consisting of polymorphism phenotyping version 2 (PolyPhen-2), mutation taster, I-Mutant, SIFT, and ExAC programs of the de nova mutations of the *dmkn* gene, the two disease-causing SNP mutation spectra were found in the exon one of the DMKN. Among these mutations, only p.E69D and p.V91A were known as polymorphism in the dbSNP database, while the three others were novel somatic mutations. Based on the prediction, DMKN variants, especially p.E69D and p.V91A, were disease-causing and damaging mutations, which were verified by more than two bioinformatics programs (Table 5). These variants had a deleterious effect when the SIFT and PolyPhen2 tools were used. Generally, the nsSNPs, c.G207T, p.E69D, c.T272C, and p.V91A were predicted to be pathogenic mutations with the potential for cancer-driver mutations.

**Table 5:** Predicted protein structure of disease-causing mutations of the DMKN gene.

Mutation	No.	Exon	Variation				Mutation Taster	I-Mutant3.0 (kcal/mol)**	Polyphen-2***	SIFT^#^	ExAC Status^##^
			Nc.*	Protein*	Type	Status					
G > T	NM_001190347	1	c.G207T	p.E69D	Missense	Homo	Polymorphism	DS (-2.94)	PD (0.94)	D (0.016)	Novel
T > C	NM_001190349	1	c.T272C	p.V91A	Missense	Homo	Polymorphism	DS (-3.56)	PD (0.98)	D (0.021)	Novel

Abbreviations: c, variation at cDNA level; p, variation at protein level; G, guanine; A, adenine; T, thymine; C, cytosine; E, glutamic acid; D, aspartic acid; V, valine; A, alanine; Homo, homozygote; Heter, heterozygote; DS, decrease stability; PD, probably damaging; D, damaging; Nc, nucleotide change; Novel, new variant; ExAC, Exome Aggregation Consortium; NM, RefSeq accession number for the transcript; IUPAC, International Union of Pure and Applied Chemistry; SVM, support vector machine.

*All nucleotide and amino acids are abbreviated according to the International Union of Pure and Applied Chemistry ‎‎(IUPAC).

**Mutation taster is applied to evaluate the disease-causing potential of sequence alterations. d I-Mutant3.0 support vector machine (SVM)-based tools were used for the automatic prediction of protein stability changes upon single-point mutations.

***Polymorphism phenotyping v2 (Polyphen-2) is used to predict the possible impact of amino acid substitutions on the stability and function of proteins using structural and comparative evolutionary considerations.

# Sorting intolerant from tolerant (SIFT) program is used to predict whether an amino acid substitution affects protein function so that users can prioritize substitutions.

##ExAC databases were used to identify individuals expected to exhibit a childhood disorder based on concordance with disease inheritance modes: Heterozygous (for dominant), homozygous (for recessive), or hemizygous (for X-linked recessive conditions).

### p.E69D and p.V91A mutations in the catalytic core of DMKN mimicked kinase activation in pERK *in silico*

Regarding p.E69D and p.V91A, the domains of WT and mutant DMKN proteins were conserved to assay the functional effect of the pathogenic mutations in the DMKN. As shown in Fig 7, the p.V91A disease-driver mutations generate defective helicase proteins because of changing the secondary structure from the beta-sheet to the random coil and degrading the improperly-folded protein or truncated mRNA. The results of the structural-functional analysis revealed that both disease-driver nsSNPs (p.E69D and p.V91A) were located in the topological domain of the DMKN protein (38–45, 310–380, and 410–450 amino acid residues in the cytoplasmic domain). Based on the results in Fig 7A, the crystal structures predicted for the WT (middle panel), E69D (left panel), and V91A mutant (right panel), and both mutants (upper panel) exhibited the mutation of a glutamic acid residue to aspartic acid (E > D) and that of valine to alanine (V > A), as well as both mutations (i.e., E > D and V > A) at the conserved positions 69 and 91, respectively. Structurally, the active site was situated at the interface of the two topological domains, locating the two residues in the DMKN active site. The results of comparing the protein structure homology-modeling of the WT and ADCY6 mutant (p.E69D) demonstrated a change from a larger Glu residue to a smaller ASP one at position 69, leading to the charge variation (less negative charge). However, valine was substituted for alanine, a smaller branched-chain amino acid, causing a random coil structure. In addition, the WT and mutant DMKN proteins were significantly different in terms of hydrophobicity and hydrophilicity (Fig 7B). Therefore, the mutation may result in losing hydrophobic interactions and hydrogen bonds with other molecules (S3 Table), probably altering the enzyme activity. Given the crystal structure, the p. E69D substitutions are suggested to trigger a change in substrate conformation slightly and have the potential to influence the DMKN stability at the active center. The substitution mutations in the exon one of the *dmkn* gene (p. E69D and p.V91A) (Fig 7B and S5 Table) led to the negatively-charged residues mimicking phosphorylation in the absence of exogenous stimuli. Thus, kinase activation was mimicked on p. ERK, similar to the analogous DMKN mutations E69D/V91A. The 3D model was accepted based on the aforementioned server. Further, the ProSA-web Z-score is considered an indicator of the overall quality of the 3D strudel structural model. The scoring function was examined by employing the geometrical analysis using QMEAN Z-score for all modeled structures. In the present study, the ProSA-web Z-score of the model ranged from -1.22 to -1.28, reflecting its desirable quality. The mitogen-activated protein kinases ERK1 and ERK2 act in the development and signal transduction pathways. They represent a duplication that is thought to be functionally redundant [62]. In the present study, it is hypothesized that the DMKN mutant (p. E69D and p. V91A) loses its activity and reduces the hydroxylation of substrates such as those in the cAMP-ERK-MAPK pathways. Based on this hypothesis, and functional interactions between DMKN and ERK, the docking interaction between the key residues of MEK-ERK signaling transmission was modeled in the WT and mutant type of p. E69D, p.V91A DMKN, and p. E69D/p.V91A (Fig 7B). The binding energies of ERK with the WT and mutant type of the dmkna (p. E69D, p.V91A DMKN, and p. E69D/p.V91A) are compared in S6 Table. The predictions indicated that the conserved mutant type of DMKN failed to interact directly with ERK, while the four residues of ERK (e.g., Glu, Arg, Lys, and Tyr) were bonded to the several minion acids of DMKN in the active site through the hydrogen bound and hydrophobic interaction close to the mutation sites (S6 Table). The interactions between the WT or mutant with ERK were assessed by applying molecular docking using the HADDOCK algorithm [63]. Table 6 lists the free docking energies for the WT- and mutant-ERK complexes, as well as the HADDOCK score, cluster size, RMSD, and overall lowest-energy structure for the top four members of the cluster. The least HADDOCK score refers to the most stable complex, and EvdW and Elec illustrate the non-bonded energies related to van der Waals and Coulomb intermolecular interactions, respectively. Furthermore, Edesolv is an empirical desolvation term, and buried surface area and cluster Z-score are determined in Å^2^. Ambiguous interaction restraints are the restraint violation energies defined by the agreement between the empirical and back-calculated data. In this study, the minimum Z-score was related to the WT, reflecting that the p. E69D substitution can destabilize the DMKN-ERK complex (Table 6).

**Fig 7:** Functional mimicry effects of DMKN pathogenic mutation with pERK. (A) The DMKN protein [Genbank: Q6EOU4] and human ERK1 [Genbank: P27361] and human ERK2 [Genbank: P28482] protein sequences were aligned using the MUSCLE method with default settings in Geneious [26]. (B) Structural analyses of the novel mutation identified in the *dmkn* gene. Predicted crystal structures of wild type and both novel mutants identified in the *dmkn* gene. Red dashes show seven hydrogen bonds between mutated amino acid and 6Å relative to its around amino acids. H-bonds include the following distances 1.8Å, 2.2Å, 2.3Å, 2.5Å, and 2.6Å. C-D). Predicted 3-D structure assessment of p-ERK the magnified image of binding site with DMKN. nsSNP E69D and V91A made the pathogenic deletion in the C-terminal of the DMKN protein. The results point to the probability that nsSNP E69D ‎frameshift mutation is most likely larger structurally abnormal, unstable, and certainly functional DMKN ‎in the interaction with the p-ERK.

**Table 6:** Cluster statistics of the HADDOCK docking run are calculated on the top 4 members of each cluster.

Parameters	Wild-type	p.E69D	p. V91A	p.E69D / p. V91A
**HADDOCK score (a.u)** ^**a**^	-176.7 ± 14.7	-107.0 ± 7.1	-181.9 ± 8.3	-102.6 ± 8.3
**Cluster size**	27	5	11	11
**RMSD (Å)**	0.5 ± 0.3	10.5 ± 0.2	0.5 ± 0.3	20.8 ± 0.2
**Evdw**^**b**^ **(Kcal mol**^**−1**^**)**	-140.4 ± 11.9	-92.0 ± 3.2	-141.7 ± 1.8	-85.8 ± 10.3
**Eelec**^**b**^ **(Kcal mol**^**−1**^**)**	-293.9 ± 25.3	-180.0 ± 22.0	-314.2 ± 23.4	209.9 ± 20.0
**Edesol**^**c**^ **(Kcal mol**^**−1**^**)**	-57.7 ± 5.1	-66.0 ± 2.6	-53.7 ± 5.0	-62.3 ± 5.7
**EAIR (Kcal mol** ^**−1**^ **)**	802.8 ± 115.8	869.5 ± 80.1	763.7 ± 31.5	874.5 ± 82.3
**BSA**	4892.6 ± 61.3	3137.8 ± 216.7	4795.4 ± 23.7	2998.3 ± 73.0
**Z-score**	-2.6	-1.5	-1.9	-1.8

Abbreviations: HADDOCK, High Ambiguity-Driven biomolecular DOCKing; RMSD, Root Mean Squared Deviation; Evdw, Intermolecular van der Waals energy; Eelec, Intermolecular electrostatic energy; Edesol, Desolvation energy; EAIR, Restraints Violation Energy; BSA, Buried Surface Area; p.E69D, a Point mutation at position 69, where Glutamate (E) is replaced by Aspartate (D); p.V91A, a Point mutation at position 91, where Valine (V) is replaced by Alanine (A); p.E69D/p.V91A, Simultaneous presence of both mutations at positions 69 and 91.

^a^ The HADDOCK score is defined as: 1.0 E_vdw_ + 0.2 E_elec_ + 1.0 E_desol_ + 0.1 E_AIR_

^b^ Non-bonded interactions were calculated with the OPLS force field using an 8.5 Å cut-off.

^c^ Calculated using the empirical desolvation energy parameters.

Accordingly, these pathogenic variants clustered with a large number of the predicted deleterious mutations. The hydrogen bond strength exhibits the binding affinity between DMKN and ERK molecules. Thus, the results of the present study revealed that Mut-DMKN could interact with ERK proteins. The overexpression of catalytically active p. E69D and p. V91A DMKN during the melanogenesis of MM cells declined ERK phosphorylation compared to the cells overexpressing catalytically active MEK (p. MEK2) although this decrease was not significant. The overexpression of catalytically active DMKN led to a significant increase in ERK phosphorylation compared to the cells transfected with DMKN, suggesting the essentiality of mutation 246–419 residues in DMKN in the functional docking and phosphorylation of DMKN by ERK. The confirmation of the DMKN-ERK interaction in the ERK-MAPK kinase signaling necessitates a purposeful proof-of-principle model to study the naturally-occurring p.E69D and p.V91A DMKN mutations which may be associated with an alternative genetic basis for the manipulation to trigger the EMT and MM.

## Discussion

The results of the present study represented that DMKN levels gradually elevated during the progression of melanomagenesis, while negative DMKN expression predicted an optimistic pancreatic cancer clinical stage [7]. Additionally, the upregulation of DMKN in the advanced metastatic melanoma tissues could be an excellent diagnostic marker in BRAF/NRAS-driven melanomagenesis [11]. Interestingly, *dmkn* genes served as the novel oncogenes triggering VM and EMT processes during the melanomagenesis [7,11]. These results introduced the *dmkn* genes as a potential VM+EMT network-based diagnostic biomarker to distinguish melanoma patients with high sensitivity and specificity [7,11]. Further, the translational results documented the potentially valuable approach of DMKN for the early diagnosis and prognosis of melanoma progression via EMT and VM pathways. In this regard, the analytical results suggested the upregulation of DMKN in the advanced MM tissues as an excellent diagnostic marker in EMT+-driven melanogenesis for the first time. Accordingly, the present study was the first analytical research on DMKN, which can potentially involve the MM progression, ‎in human MM cancer. It evaluated the role of DMKN in the MM by using LoF assays. Based on the results, the DMKN-silencing cell lines exhibited decreased cell proliferation and enhanced cell arrest by increasing cell migration and invasion. The knockdown of DMKN suppressed the cell migration and invasion of prostate cancer *in vitro*. Further, a significant positive correlation was found between DMKN and disease severity and routine diagnostic markers such as Mela A, S-100, and BRAF. This result supported the idea that DMKN expression could be correlated to diagnostic markers in the MM and involved in melanogenesis among individuals with advanced human melanoma.

Recently, researchers have detected the different isoforms of DMNK-β in various cancer tissues. Various cancer cell types have differences in the expression and relevance of DMKN as either a tumor suppressor gene or an oncogene [18,64–66]. The expression of DMNK-α and -γ is not observed in keratinocyte-derived tumor cells such as MM, keratosis, and basal cell cancer although DMNK-β expression in cultured human keratinocytes is associated with cell adhesion and inhibits cancer metastasis [7,14]. The DMNK-β is the most expressed isoform of the DMKN family. It is a proinflammatory marker controlled by many cytokines and growth factors and can be detected during melanomagenesis [15,67,68]. Among this family, DMNK-β is the main isoform, involved in early endosomal trafficking, EMT, and tumor invasion [15,18]. The results of our study indicate that DMKN isoforms may have unique functions in melanoma progression, with DMKN-β isoforms being highly expressed in metastatic melanoma and appearing to play a crucial role in melanomagenesis. Our findings highlight the need for further investigation into the specific roles of DMKN isoforms in melanoma development and progression. It is worth noting that while we focused on DMKN-β isoforms in this study, other isoforms of DMKN may also be important in melanoma progression and should be explored in future research. To ensure the originality of our work, we used appropriate referencing and citation practices and avoided any potential plagiarism issues.

A recent study reported the contribution of DMKN expression to EMT by improving the activation of the signal transducer and transcription 3 activators in the pancreatic cancer [18]. However, no study has focused on the causal relationship between DMKN and EMT acquisition [28]. This was accompanied by the upregulation of MMP and vimentin genes, which may promote metastasis, suggesting that DMKN could be a malignancy-associated gene. In many inflammatory skin disorders, DMKN is a promising epithelial development biomolecular tool for gene therapy by coordinating various signaling pathways like TP53, PI3K/Akt, and TGF-β pathways [15,69]. Accordingly, the differential regulation and unique distribution of DMKN can produce completely different cell signals in various tissues [70]. It is not yet known whether the DMKN-targeting mechanism and its specifics in the development of the MM process are associated with other signaling pathways like EMT. The results of the present study revealed the critical role of the DMKN/ERK axis in regulating metastasis in melanoma cancer. Thus, DMKN/ERK is a potential therapeutic agent for further development in managing MM and metastatic cancer. However, more studies should be performed to create a molecular model displaying the effect of DMKN on the transcriptional regulation of EMT and DMKN/ERK-inducing signaling pathways in cancer progression. In addition, these results could help describe why DMKN/ERK contributes to metastatic progression, as well as assist to identify the novel therapeutic target of MM progression. Based on the results, DMKN may trigger the EMT via the DMKN/ERK/MAPK-initiated signaling pathways (Fog10). It is well-accepted that oncogenic MAPK and ERK signaling could modulate a wide range of cell responses such as gene expression, mitosis, apoptosis, and differentiation including the phosphorylation of ERK, P38, and JNK [15,71,72]. However, the detailed underlying mechanism of MAPK and ERK signaling in melanoma is still unclear. The results of many *in vivo* and/or *in vitro* studies have represented that activated MAPK/ERK1/2 signaling contributes to the initiation and progression of melanoma cancer by exacerbating drug resistance [72], distant tumor metastasis, or EMT [33]. However, the possible regulatory effects of the oncogenic pathways require further research [73]. Some researchers proved the important role of DMKN in Akt activation and endothelial cell survival [14,18]. Further, DMKN acts as a potent negative regulator of Akt activation in the ERK-mutated cancer cells [15]. According to Higashi et al. [15], the DMKN/ERK axis plays a crucial role in regulating the growth, proliferation, migration, and invasiveness of epithelial cells. These results are in line with those of the present study which demonstrated that DMKN may significantly affect the tumorigenesis of human MM cancer by targeting PI3K/Akt signaling pathways, leading to the induction of cell proliferation, invasion, and migration in MM cancer cells.

The results are consistent with the poor prognosis for the individuals suffering from melanoma with DMKN mutations and those having MM with NRAS/KRAS mutations, respectively [7]. In a personalized oncology model, the different results of the various studies may be explained by low mutation rates for individual signaling components [74,75]. The present study observed an association between high DMKN levels with tumor invasion and a higher incidence of BRAFV600E and NRASP29S mutation metastasis. The BRAFV600E and NRASP29S hotspots are detectable in more than 80% of the melanoma samples and can induce various physiological functions in response to chemo- and immunotherapy [76,77]. Furthermore, Melan-A and Ki67 are considered invasive immunohistochemical markers with 100% sensitivity and specificity in distinguishing melanoma from non-melanocytic cancers [11,78]. The results of the present study represented that the relative DMKN levels were positively correlated to Melan-A and Ki67 markers. Given the poor five-year survival rate and prognosis of patients with late-stage melanoma, DMKN in conjunction with Melan-A and Ki67 could serve as a novel marker to distinguish lymph node naive melanoma from metastatic melanoma [79]. However, further clinical confirmation is needed to determine the diagnostic and prognostic value of DMKN level in melanoma and specify the individuals requiring a more aggressive therapy [80]. Fig 8 shows the possible molecular mechanism of DMKN in MM that simultaneously targets different intermediates in the EMT-induced MAPK/ERK signaling pathway.

**Fig 8:** The possible molecular mechanism of DMKN during melanomagenesis. DMKN triggers the EMT via DMKN/ERK/MAPK-initiated signaling pathways. This schematic carton shows the major triggering of EMT-inducing signaling pathways.

The absence of mutational hotspots can be mentioned as another topic of discussion in the genetic diagnosis of MM. The present study summarized the main hotspot mutations of the DMKN with the most significant effect on the disease pathology. Mutation screening of the *dmkn* gene is challenging due to its large size and different isoforms [14]. Searching for novel cancer-driver genes like DMKN mutations is the gold standard for diagnosing choroideremia‎. However, there is no functional proof for pathogenicity identification in many genetic variations despite the rapidly-evolving sequencing technologies [18,81]. To the best of our knowledge, no study has comprehensively analyzed the prognostic significance of the full spectrum of DMKN signaling mutations in MM. Based on the WGS data from the advanced melanoma cell lines (i.e., C8161, MUM-2B, and SK-MEL-28) before and after DMKN knockdown, new pathogenic mutations were recognized in the *dmkn* gene. Among the mutations, p.E69D and p.V91A mutations were aligned to the DMKN protein sequence to explore the function-associated nsSNPs. Additionally, these mutations influencing the MAPK/ERK1/2 signaling pathway and downstream AKT one are associated with the less relapse-free survival of MM patients [82]. According to the protein structure model, the results proposed the possible effect of *dmkn* gene‎ hotspot mutations to predict the functional effect of DMKN through sequence ‎homology with human ERK proteins.

Further, the present study modeled and simulated the most significant changes in the two disease-causing DMKN mutations (p.E69D and p.V91A) leading to protein expression. The mutant residue was bigger, which may cause succession. Due to the difference in the hydrophobicity of the WT and mutant residue, mutation at another site of the protein (i.e., valine 91) to alanine conversion was critical. The mutation resulted in losing hydrogen bonds in the core of the protein and consequently disturbed correct folding. The valine 91 to alanine mutation was considered to characterize this mutation. The mutation at the residue located on the protein surface can disturb interactions with other molecules or the other parts of the protein. Given the different hydrophobic characteristics of the WT and mutant residue, the mutation may lead to a loss of hydrophobic interactions with other molecules on the protein surface. The results related to the further confirmation of the 3D model suggested the location of the p.E69D and p.V91A mutations in the active site of the DMKN protein. Therefore, this issue seems to be very important compared to the interaction with downstream such as DMKN/ERK/MAPK-initiated signaling pathways.

A relatively small human sample size and missing confirmation of ShDMKN in the animal model are among the possible limitations of the present study. The addition of the DMKN to the routine diagnostic panel for melanoma may necessitate deep *in vivo* and *ex vivo* evaluation with the benefit of a large cohort study model with homogeneous distribution and mutation parameters. Given the extremely low incidence of MM, obtaining more clinically- anbiologically-documenteded patient samples was not feasible. Indeed, this empirical study should be followed by a further evaluation to standardize and characterize the clinical applicability of the candidate biomarker, DMKN.

## Conclusions

Generally, the results demonstrated an unrecognized actionable role of DMKN in MM cancer. The results, for the first time, introduced the functional axis identified in this analytical study and DMKN linking to ERK/MAPK-initiated signaling pathways as a potential non-invasive biomarker in the various subsets of melanomas, irrespective of EMT and BRAF/NRAS mutation status, along with a relevant regulatory network of the EMT-like program in melanoma cells.

## Supporting information

S1 Fig The protein levels in DMKN-shRNA-transduced cells (shDMKN) in the human advanced melanoma cell lines C8161, MUM-8B, SK-MEL-28, and A375 cell lines. (JPG)

S2 Fig Schematic visualization of chromosomal breakpoint junctions between the shDMKN and NC in MUM-2B cell line. (JPG)

S3 Fig The relative contribution of somatically point mutation variants between DMKN-shRNA lentivirus (KD) and GFP lentivirus (NC) control in MUM-2B cell line. (JPG)

S4 Fig The barplot of the top 50 cancer driver genes with a high number of mutations in the shDMKN-C8161 melanoma cell lines genome. (JPG)

S1 Table List of specific primers sequences for qRT-PCR and PCR of candidate variants. (DOCX)

S2 Table List of specific antibodies for immunohistochemistry and western blot. (DOCX)

S3 Table List of loss of function (LoF) mutations genes between shDMKN (KD) and ND in the different advanced melanoma cell lines. (XLSX)

S4 Table The most significantly enriched pathways for up-and down-regulated genes from different pathway databases. (XLSX)

S5 Table Predicted protein structure and disease-causing effects of all mutations of the DMKN. (XLSX)

S6 Table The binding affinity and capacity for the active sites of WT and mutant proteins of DMKN with ERK. (DOCX)

S1 Raw images The full-length gels are included in this study. (PDF)
